The article "Transplantation of HGF gene-engineered skeletal myoblasts improve infarction recovery in a rat myocardial ischemia model" was retracted in 2023. Reasons: duplicated images; overlap with earlier publications; unreliable data; concerns about the images.

# Transplantation of *HGF* gene-engineered skeletal myoblasts improve infarction recovery in a rat myocardial ischemia model

**DOI:** 10.1371/journal.pone.0175807

**Published:** 2017-05-01

**Authors:** Shu-Ling Rong, Xiao-Lin Wang, Cui-Ying Zhang, Zhuo-Hui Song, Lu-Hua Cui, Xiao-Feng He, Xu-Jiong Li, Hui-Jin Du, Bao Li

**Affiliations:** 1 Department of Cardiology, Heping Hospital and Institute of cardiovascular disease, Changzhi Medical College, Changzhi, China; 2 Department of Cardiology, The Second Hospital of Shanxi Medical University, Taiyuan, Shanxi, China; 3 Department of Pediatrics, Heping Hospital and Institute of cardiovascular disease, Changzhi Medical College, Changzhi, China; 4 Department of Physiology, Changzhi Medical College, Changzhi, China; 5 Department of Research, Heping Hospital, Changzhi Medical College, Changzhi, China; Indiana University School of Medicine, UNITED STATES

## Abstract

**Background:**

Skeletal myoblast transplantation seems a promising approach for the repair of myocardial infarction (MI). However, the low engraftment efficacy and impaired angiogenic ability limit the clinical efficiency of the myoblasts. Gene engineering with angiogenic growth factors promotes angiogenesis and enhances engraftment of transplanted skeletal myoblasts, leading to improved infarction recovery in myocardial ischemia. The present study evaluated the therapeutic effects of hepatocyte growth factor (*HGF*) gene-engineered skeletal myoblasts on tissue regeneration and restoration of heart function in a rat MI model.

**Methods and results:**

The skeletal myoblasts were isolated, expanded, and transduced with adenovirus carrying the *HGF* gene (Ad-HGF). Male SD rats underwent ligation of the left anterior descending coronary artery. After 2 weeks, the surviving rats were randomized into four groups and treated with skeletal myoblasts by direct injection into the myocardium. The survival and engraftment of skeletal myoblasts were determined by real-time PCR and *in situ* hybridization. The cardiac function with hemodynamic index and left ventricular architecture were monitored; The adenovirus-mediated-*HGF* gene transfection increases the HGF expression and promotes the proliferation of skeletal myoblasts *in vitro*. Transplantation of *HGF*-engineered skeletal myoblasts results in reduced infarct size and collagen deposition, increased vessel density, and improved cardiac function in a rat MI model. *HGF* gene modification also increases the myocardial levels of HGF, VEGF, and Bcl-2 and enhances the survival and engraftment of skeletal myoblasts.

**Conclusions:**

*HGF* engineering improves the regenerative effect of skeletal myoblasts on MI by enhancing their survival and engraftment ability.

The article "Transplantation of HGF gene-engineered skeletal myoblasts improve infarction recovery in a rat myocardial ischemia model" was retracted in 2023. Reasons: duplicated images; overlap with earlier publications; unreliable data; concerns about the images.

## Introduction

Although various approaches have greatly advanced in the diagnosis and treatment of cardiovascular diseases, heart failure remains the leading cause of mortality in elderly patients [1]. The major pathophysiological features for mortality caused by chronic heart failure (CHF) include left ventricular (LV) dysfunction and heart remodeling post-infarction. Current treatments including the intervention or pharmacological therapies have achieved limited success in the treatment of CHF owing to their inefficient recovery of the infarcted heart.

Cell therapy is emerging as a promising regenerative approach to treating all stages of heart failure following myocardial infarction (MI) [2]. Hitherto, several cell types, such as embryonic stem cell-derived cardiomyocytes, mesenchymal stem cells, and skeletal myoblasts, have been shown to successfully prevent or reverse the vascular injury and LV remodeling post-MI [3–5]. However, the functional benefits of cell therapy in CHF are proportional to cell engraftment [6]. Thus, several strategies including physiological pretreatment, anti-apoptosis, and angiogenic gene transfection have been evaluated for improving the cell engraftment [6–9].

The combination of gene and cell therapy has demonstrated a synergistic effect valuable in improving the cell engraftment in ischemic myocardium [10]. Transfection with anti-apoptotic genes such as *Bcl-2*, thioredoxin-1 (*Txn-1*), and *Akt* enhances cell survival, leading to improved functional benefits of cell transplantation [11–13]. Furthermore, cells engineered with angiogenic growth factor genes could induce therapeutic angiogenesis, increase perfusion, and improve the heart function post-MI in animal models [14, 15]. The transplantation of skeletal myoblasts has been undertaken as a novel therapeutic option to regenerate the infarcted myocardium. However, the use of myoblasts alone limits the treatment of CHF due to the insufficient expression of angiogenic growth factors and low engraftment ability after transplantation. Engineering with angiogenic growth factors, such as colony stimulating factor-1, is a state-of-the-art strategy to improve the therapeutic success of skeletal myoblasts in the treatment of MI [16].

Hepatocyte growth factor (HGF) is an angiogenic growth factor with multiple functions including angiogenesis, mitogenesis, morphogenesis, and organ regeneration activities in a wide variety of cells [17]. HGF has been shown to play a major role in therapeutic angiogenesis, cardioprotection as well as tissue regeneration after MI [18]. Gene therapy based on *HGF* results in therapeutic angiogenesis and decreased apoptosis, thereby, leading to the regeneration of endothelial cells and myocardiocytes in the infarcted myocardium. Furthermore, HGF-engineered cell therapy has emerged as a novel approach to promoting therapeutic angiogenesis and tissue regeneration in critical limb ischemia [19]. Both experimental and preliminary investigations have demonstrated the feasibility and efficacy of *HGF* gene therapy in the treatment of ischemic heart diseases [20, 21].

The article "Transplantation of HGF gene-engineered skeletal myoblasts improve infarction recovery in a rat myocardial ischemia model" was retracted in 2023. Reasons: duplicated images; overlap with earlier publications; unreliable data; concerns about the images.

Skeletal myoblasts and *HGF* gene transfer promote angiogenesis, reduce the myocardial fibrosis, and protect the cardiomyocytes from apoptosis [21–23]. However, the synergistic effects and mechanisms underlying the skeletal myoblasts engineered with *HGF* to treat acute MI (AMI) remain unknown. In the present study, we transduced skeletal myoblasts with adenoviral vectors carrying the *HGF* gene and evaluated their therapeutic effect on MI in a rat model.

## Materials and methods

### Experimental animals

Sprague–Dawley (SD) rats were obtained from the Animal Center of Academy of Military Medical Science (Beijing, China) and used as cell donors or recipients, respectively. The Institutional Animal Care and Use Committee of the Changzhi Medical College approved all the experiments in this study. The rats were housed in a clean environment with 12 h light-dark cycle at 25°C and 40–70% humidity and fed standard laboratory chow and water ad libitum. During the experimental procedures, the animals were weighed daily and monitored for any change in the behavior, food or water consumption, infection, and mortality. The male neonatal rats (1–3-day-old) were sacrificed to obtain skeletal myoblasts that were cultured, and 10–12-week-old female rats underwent surgery for the cell transplantation. In addition, we also utilized an approved protocol for the early euthanasia/humane endpoints in animals that became severely ill during the experiment. Such rats were euthanized by carbon dioxide (CO_2_) asphyxiation. Clinical symptoms, including rapid weight loss, loss of appetite for more than 3 days, extremely weakened to access water and food, an infection that did not respond to drug therapy, were used as markers to determine the appropriate point in time for euthanizing the animals.

### Isolation and culture of skeletal myoblasts

Primary skeletal myoblasts were isolated and cultured from male neonatal SD rats as described previously [24, 25]. Briefly, the primary skeletal myoblasts were isolated from the hind limb muscles of neonatal SD rats (1–3-day-old). The muscles were dissected from the connective tissues, minced into pieces of approximately 1 mm^3^ and treated with 0.25% trypsin (Gibco, USA) at 37°C for 1 h. The samples were filtered through the nylon mesh and centrifuged at 1000 rpm for 3 min to separate the dissociated cells. The pellet was resuspended in DMEM growth medium supplemented with 20% fetal bovine serum (FBS) and dispensed in culture dishes. The cells were incubated at 37°C in the presence of 5% CO_2_. The purity of primary skeletal myoblasts was evaluated by immunocytochemistry staining method with monoclonal antibodies against Desmin (1:500, Santa Cruz Biotechnology, USA). The Desmin-positive cells in five randomly selected areas of each culture dish were counted under a microscope. The skeletal myoblasts at passage 3 were used for *b*oth *in vitro* and *in vivo* studies.

The article "Transplantation of HGF gene-engineered skeletal myoblasts improve infarction recovery in a rat myocardial ischemia model" was retracted in 2023. Reasons: duplicated images; overlap with earlier publications; unreliable data; concerns about the images.

### Adenoviral vectors and gene transfection

The adenovirus carrying the *HGF* gene (Ad-HGF) and control adenovirus (Ad-GFP) were a kind gift from the Beijing Institute of Radiation Medicine. These recombinant replication-deficient adenoviruses were amplified in HEK293 cells and purified by ultracentrifugation on a cesium chloride gradient. The final plaque-forming units (pfu) were determined by titrating the HEK293 cells by the agarose overlay method. The skeletal myoblasts were infected with the recombinant adenovirus at an MOI (multiplicity of infection) of 150. Subsequently, the efficiency of infection was determined by the percentage of GFP+ cells in Ad-GFP-transduced skeletal myoblasts.

### Immunocytochemistry, real-time quantitative PCR (RT-PCR), enzyme-linked immunosorbent assay (ELISA)

Skeletal myoblasts (2×10^6^ cells/dish) transduced with Ad-HGF (SM-HGF group)or Ad-GFP (SM-GFP group) were cultured. Immunocytochemistry examines the surfaced expression of HGF in the skeletal myoblasts. These cells were stained with anti-human HGF monoclonal primary antibody (Santa Cruz Biotechnology, USA), followed by the appropriate HRP-linked secondary antibody. Cells were visualized under a microscope.

The mRNA levels of *HGF* and *GAPDH* genes in skeletal myoblasts transfected with Ad-HGF and Ad-GFP were estimated on day (D) 3 post transfection by RT-PCR as described previously [24, 25]. Briefly, the total RNA was extracted by TRIzol, and 1 μg total RNA was subjected to reverse transcription of mRNA to cDNA using a Reverse Transcription System Kit (Promega, USA) according to the manufacturer’s protocols. The primer sequences and PCR product length of human *HGF* and *GAPDH* were listed in Table 1 [26]. The band intensity of each gene was quantified on agarose gels using densitometry, and the ratio of *HGF* to *GAPDH* genes was used for a semi-quantitative estimation of gene expression.

**Table 1:** PCR primer sequences of *GAPDH*, h*uman HGF*, *Sry* genes.

Gene	Primer
*GAPDH*	
Forward	5’-TGAAGGTCGGAGTCAACGGATTTGGT-3’
Reverse	5’-CATGTGGGCCATGAGGTCCACCAC-3’
*HGF*	
Forward	5’-AAA TGC AAA CAG GTT CTC AAT GT-3’
Reverse	5’-ATG CTA CTC GGA CAA AAA TAC CA-3’
*Sry*	
Forward	5’-CATCGAAGGGTTAAAGTGCCA-3’
Reverse	5’-ATAGTGTGTAGGTTGTTGTCC-3’

The HGF in the culture supernatant was also assessed by ELISA Kit (R&D Systems Inc., USA) according to the manufacturer’s protocols.

The article "Transplantation of HGF gene-engineered skeletal myoblasts improve infarction recovery in a rat myocardial ischemia model" was retracted in 2023. Reasons: duplicated images; overlap with earlier publications; unreliable data; concerns about the images.

### Cell proliferation *in vitro*

2 ×10^6^ skeletal myoblasts of the three groups (SM-HGF group, SM-GFP group, and cell control group) were cultured and passaged. On D3, D7, and D14 after transfection, the cell number was counted. The increase in cell number calculated between D3 and D14 was considered as an index of cell proliferation.

### Rat MI model and treatment

10–12-week-old female SD rats were used. MI was induced by ligating the left anterior descending coronary artery as described previously [24, 25]. Briefly, a small thoracotomy was carried out through the left fourth intercostal space, and then, the left anterior descending coronary artery of the rat was ligated by a 6–0 surgical suture. The antibiotics and buprenorphine hydrochloride were administered after the operation. 16/80 (20%) rats perished within 2 weeks after the coronary artery ligation surgery. 4/16 rats did not wake up after the surgery and deceased as a result of technical surgical failure on D0 of surgery. Surprisingly, 5 rats died from D2–D9 post-operation. Seven rats were euthanized by CO_2_ asphyxiation because of rapid weight loss, weakened ability even for access to water and food, and infection that did not respond to drug therapy on D2–D13 post-operation. Surviving rats that underwent ligation were randomly divided into four groups 2 weeks after the left coronary artery occlusion. These rats underwent transplantation of skeletal myoblasts transduced with Ad-HGF (SM-HGF group), with Ad-GFP (SM-GFP group), or non-transduced (SM group). A control group was administered only the culture medium. The SM-HGF, SM-GFP, SM only, and medium were injected into the border zone surrounding the infarct (injections of 5x10^6^ cells in 150 μL serum-free culture medium) with a 27G needle. The sham rats (sham group) underwent a sham operation comprising of thoracotomy and cardiac exposure but without coronary artery ligation. Surprisingly, 2 weeks after cell transplantation, 2 rats from the control group died probably due to a thoracic infection that was unresponsive to drug therapy; no mortality was recorded in the groups that received cell therapy.

### Determination of cell survival *in vivo*

One week after cell transplantation, the transplanted area was harvested, the frozen LV samples were sliced into 6-μm sections, and the GFP+ cells in the transplanted area were observed by fluorescence microscope. The site was also stained with hematoxylin and eosin (HE) method. The rate of cell survival in female rats was detected using the Y chromosome RT-PCR after 1 and 4 weeks treatment. Briefly, genomic DNA was isolated from the transplanted area in each of the three groups. The DNA was dissolved in 100μL of water, and the amount and purity of the DNA were measured by Spectrophotometer. The DNA samples were amplified by real-time PCR. The assay was analyzed by the ABI 7300 Real-Time PCR System (Applied Biosystems, Foster City, CA, USA). The standard curve was created by mixing 0, 10, 100, 1,000, 10,000, and 100,000, male myoblasts into diluted homogenate of female ventricles. The primer sequences and the length of the PCR product of male rat *Sry* gene on the Y chromosome were listed in Table 1 [27].

The article "Transplantation of HGF gene-engineered skeletal myoblasts improve infarction recovery in a rat myocardial ischemia model" was retracted in 2023. Reasons: duplicated images; overlap with earlier publications; unreliable data; concerns about the images.

Subsequently, after 4 weeks, the *in situ* hybridization for *Sry* gene was utilized for identifying the implanted cells in the ischemic myocardium. The sections were mounted on silanized slides and dried overnight at 60°C. Then, the slides were deparaffinized, hydrated, and incubated in 3% hydrogen peroxide in PBS for 30 min to quench the endogenous peroxidase. The sections were treated with 0.5% pepsin for 10 min at 37°C. After rinsing with 0.1X PBS, the sections were placed in a boiling water bath for 15 min and rapidly cooled on ice, followed by overnight hybridization with DIG-labeled probes at 42°C overnight. Subsequently, the sections were washed and blocked with Blocking Reagent (Roche Diagnostics, Switzerland). Finally, DIG was detected with anti-DIG antibody conjugated with alkaline phosphatase (Roche Diagnostics), the slides were washed with maleic acid buffer, and color-developed using BCIP/NBT (Roche Diagnostics).

### ELISA and Western blot

The HGF in the transplanted area was assessed by ELISA. The cell implanted area was harvested and lysed at 1 week after transplantation. The levels of HGF and VEGF were assessed using commercially available ELISA Kits according to the protocols recommended by the manufacturer.

One week after cell transplantation, the levels of Bcl-2 protein in the transplanted scar area were estimated by Western blot. Tissue samples from the transplanted area were dissected and homogenized in the lysis buffer to prepare the whole protein extract. Equivalent amounts of proteins were separated by sodium dodecyl sulfate-polyacrylamide gel electrophoresis (SDS-PAGE), transferred to nitrocellulose membranes and probed with an anti-rat Bcl-2 polyclonal antibody (Santa Cruz Biotechnology). After washing and incubating with horseradish peroxidase (HRP)-conjugated secondary antibody, the immunoreactive bands were visualized using ECL detection reagents. The proteins levels of Bcl-2 were estimated after normalizing against the β-actin internal control.

The article "Transplantation of HGF gene-engineered skeletal myoblasts improve infarction recovery in a rat myocardial ischemia model" was retracted in 2023. Reasons: duplicated images; overlap with earlier publications; unreliable data; concerns about the images.

### Cardiac function studies

Hemodynamic studies were performed 4 weeks after treatment. After anesthetizing the animals with pentobarbital, followed by intubation, a catheter was inserted first into the right carotid artery and then into the left ventricle. The hemodynamic variables were measured with a pressure transducer connected to a PowerLab system (AD Instruments, Australia). LV systolic pressure (LVSP), LV end-diastolic pressure (LVEDP), and the maximal and minimal first derivatives (LVdP/dt_max_ and LVdP/dt_min_) were measured.

### Infarct size, collagen deposition, and vessel density

After completing the hemodynamic measurements, the hearts of all the rats were arrested in diastole by intravenous injection of 2–3 mL 10% KCl. The hearts were removed, perfused with PBS, and frozen immediately. Transverse sections for every 2 mm of the left ventricle were cleaved, and the slices were fixed in 10% phosphate-buffered formaldehyde. The paraffin-embedded tissues were sectioned into 4-μm-thick slices. These sections were subjected to HE staining. Digital images for epicardial and endocardial circumferences, areas, LV free wall, and infarct size were captured by Scion Image software and assessed. The infarct size in each heart was calculated as the percentage of infarct scar relative to the outer circumference of the LV free wall. The non-infarcted areas were stained with collagen-specific Sirius Red stain. The sections were incubated with anti-rat type I collagen primary antibody, followed by the biotinylated secondary antibody. The image of each field of non-infarcted myocardium was acquired, and the area of interstitial fibrosis was calculated as the ratio of the total area of interstitial fibrosis to the total area of connective tissue.

The vascular density in the implanted region of the hearts (n = 6/group) was evaluated 4 weeks after cell transplantation. The fixed tissues were sectioned and stained with antibodies against factor VIII (Maixin-Bio, China) to facilitate the quantification of vascular density in the border zone. The number of vessels per high-power field was counted by two blinded observers in five fields per slide; the mean of vessels/field was used for subsequent analysis.

### Statistical analysis

Data are expressed as mean ± SEM. The differences in the quantitative data and between the groups were assessed by the paired sample t-test and one-way analysis of variance (ANOVA), respectively. SPSS 13.0 software was used for all analyses. P<0.05 was considered as significant difference.

The article "Transplantation of HGF gene-engineered skeletal myoblasts improve infarction recovery in a rat myocardial ischemia model" was retracted in 2023. Reasons: duplicated images; overlap with earlier publications; unreliable data; concerns about the images.

## Results

### Isolation and characterization of skeletal myoblasts

The neonatal SD rats were used to isolate the skeletal myoblasts. The morphology of the skeletal myoblasts in primary culture was illustrated in Fig 1A immunocytochemistry staining using Desmin antibody. As shown in Fig 1B, more than 98% skeletal myoblasts were positive for Desmin. The Desmin proteins were localized primarily in the cytoplasm of the skeletal myoblasts.

**Fig 1:** Identification of myoblasts by immunocytochemistry. (a) Representative images of myoblasts at day 4 after the primary culture (original magnification ×200). (b) Immunocytochemistry staining of myoblasts by Desmin antibody. Desmin is observed in the cytoplasm (SP, original magnification ×400).

### Adenovirus-mediated HGF expression in skeletal myoblasts

To optimize the efficiency of adenovirus infection in skeletal myoblasts, we compared the percentage of GFP+ skeletal myoblasts transfected with Ad-GFP at different MOIs. Fig 2A showed that high transfection efficiency and low toxicity could be achieved in skeletal myoblasts by Ad-GFP at an MOI 150. Therefore, the myoblasts were transfected with Ad-HGF at MOI 150 in the subsequent experiments.

**Fig 2:** Adenovirus-mediated HGF expression in skeletal myoblasts. (a) GFP expression in myoblasts transfected with Ad-GFP by fluorescence microscopy (original magnification ×400); (b) Immunocytochemistry staining for human HGF in myoblasts transfected with Ad-HGF (immunocytochemistry staining, original magnification ×400). (c) Immunocytochemistry staining in untransfected control myoblasts (immunocytochemistry staining, original magnification ×400). (d) RT-PCR-based assessment of human *HGF* gene in myoblasts transfected with Ad-HGF. (e) The RT-PCR analysis of HGF mRNA in SM infected with Ad-HGF, Ad-GFP, and SM only. (f) The Ad-HGF-transduced myoblasts were cultured for 14 days. The conditioned medium was collected at different points in time, and the HGF protein was determined by ELISA. Significant differences were found in myoblasts infected with Ad-HGF (SM-HGF group) as compared to myoblasts infected with Ad-GFP (SM-GFP group) and non-infected myoblasts (SM group) (n = 6, P<0.05, *P<0.05 *vs*. SM group control cell; #P<0.05 *vs*. SM-GFP group).

The skeletal myoblasts were transduced with Ad-GFP (SM-GFP group) and Ad-HGF (SM-HGF group), respectively. The expression of HGF was determined by immunocytochemistry, RT-PCR, and ELISA. The results showed that the positive staining by HGF antibodies was observed in the Ad-HGF-infected group (Fig 2B); a similar result was not observed in the untransfected myoblasts (Fig 2C). A 454 bp-specific PCR product of human HGF was observed in the Ad-HGF-transduced skeletal myoblasts but not in cell control group (SM group) and SM-GFP group (Fig 2D). Furthermore, the human HGF mRNA was detected by RT-PCT in the SM-HGF group (Fig 2E). The protein content in the supernatant from the culture of Ad-HGF-transduced skeletal myoblasts was determined by ELISA, which revealed that the HGF concentration in the Ad-HGF-infected group peaked at 2 days post-infection and was maintained at a high level for a minimum of 2 weeks (Fig 2F).

The article "Transplantation of HGF gene-engineered skeletal myoblasts improve infarction recovery in a rat myocardial ischemia model" was retracted in 2023. Reasons: duplicated images; overlap with earlier publications; unreliable data; concerns about the images.

### Ad-HGF transfection enhances the proliferation of myoblasts *in vitro*

The skeletal myoblasts transduced with Ad-HGF or Ad-GFP were assayed for proliferation. 2×10^6^ cells were seeded and cultured for 14 days; the cell numbers on D3, D7, and D14 were calculated. Fig 3A displayed the morphology of Ad-HGF-transduced skeletal myoblasts on D3 and D7 post-transfection. As shown in Fig 3B, the numbers of cells in the SM-HGF and SM-GFP groups, were significantly lower than that in the SM group at D3 post-transfections (1.31 ± 0.10 ×10^6^ and 1.33 ± 0.09 ×10^6^ *vs*. 2.65 ± 0.13 ×10^6^ cells, n = 6). However, the cell numbers in the SM-HGF group, SM-GFP group, and control group increased to 11.1 ± 1.09×10^6^, 7.8 ± 1.1×10^6^, and 10.0 ± 1.03 ×10^6^ cells on D14 post-transfection. The expansion rate of SM-HGF group was found to be higher than that of the control group (Fig 3C).

**Fig 3:** Ad-HGF transfection enhances the proliferation of skeletal myoblasts. (a) The morphology of skeletal myoblasts transduced with Ad-HGF cultured for 3 (left) and 14 (right) days. (b) The myoblasts were transduced with Ad-HGF and control vector, respectively. 2x10^6^ cells were seeded and cultured for 14 days. The cell numbers were counted at different points in time. (c) The expansion rate of myoblasts in the culture at day 14 post-transfection (n = 6, P<0.05, *P<0.05 *vs*. SM group control cell; ^#^P<0.05 vs. SM-GFP group).

### HGF modification increases the survival and engraftment of skeletal myoblasts

One week after cell implantation, the GFP+ cells were observed in frozen LV samples by fluorescence microscopy. Fig 4A demonstrated that the GFP+ cells surrounded the myocardial scar tissue, indicating the survival of SM-GFP cells. The myocardium was shown by HE staining (Fig 4B).

**Fig 4:** Assessment of engraftment and cell survival after cell transplantation. One week after cell transplantation, the GFP+ cells in frozen LV samples (SM-Ad-GFP group) were observed by fluorescence microscope (a). The left myocardium was stained with HE and observed in the bright-field (b). The number of surviving cells (detected using Y chromosome real-time PCR) in the myocardial at week 1 (c) and week 4 (d) after cell transplantation (n = 6, P<0.05, *P<0.05 *vs*. SM group control cell; ^#^P<0.05 *vs*. SM-GFP group). The *Sry* gene-positive cells were identified within the transplanted area in all groups with the use of in situ hybridization 4 weeks after cell transplantation (Fig 4E). The arrows showed the *Sry*-positive cells.

The article "Transplantation of HGF gene-engineered skeletal myoblasts improve infarction recovery in a rat myocardial ischemia model" was retracted in 2023. Reasons: duplicated images; overlap with earlier publications; unreliable data; concerns about the images.

One week and 4 weeks after cell implantation, the number of surviving cells harboring the Y chromosomes, as detected by RT-PCR, was greater (P<0.05, n = 6/group) in the HGF-transfected group as compared to the SM-GFP group and SM group (Fig 4C and 4D), respectively.

After 4 weeks, *Sry* gene-positive cells were identified within the transplanted area in all groups by *in situ* hybridization (Fig 4E). The number of grafted cells (*Sry* gene-positive cells) was significantly higher in the SM-HGF groups as compared to the SM-GFP and SM groups (P<0.05, n = 6/group), respectively.

### Implantation of Ad-HGF-transduced myoblasts increases HGF, VEGF, and Bcl-2 expression in myocardium

The HGF expression in the tissue lysate from the injected area in the SM-HGF group was determined by ELISA. The level of HGF protein in the SM-HGF group was significantly higher than that in the SM-GFP and cell-only groups (Fig 5A). Since HGF induces therapeutic angiogenesis via generation of VEGF in skeletal muscle cells, the level of VEGF protein in SM-HGF injection areas was also determined [17, 28]. The implantation of SM-HGF cells increased the level of VEGF in myocardial tissues (Fig 5B). In addition, the ratio of Bcl-2 to β-actin in the transplanted area was greater in the HGF groups as compared to both vector and cell groups (P<0.05, n = 6/group,).

**Fig 5:** Implantation of HGF-modified skeletal myoblasts increases the HGF and VEGF expression in the myocardium. The Ad-GFP- or Ad-HGF- transduced myoblasts were implanted into the myocardium in an MI model for 7 days. The protein levels of HGF (a) and VEGF (b) in the transplanted area were determined by ELISA. (c) Western blot was performed for Bcl-2 expression in SM transduced with Ad-HGF, vector control, and cell control group. (d) The ratio of Bcl-2 to β-actin in the transplanted area was evaluated by Western blot (n = 6, P<0.05, *P<0.05 *vs*. SM group; ^#^P<0.05 *vs*. SM-GFP group, ^†^P<0.05 *vs*. control group).

### Implantation of HGF-engineered skeletal myoblasts improves heart functions

The skeletal myoblasts transduced with Ad-GFP and Ad-HGF, respectively, were implanted into the ischemic myocardium. The functional parameters of the heart were determined at week 4 after cell transplantation. The implantation of HGF-transduced myoblasts improved the cardiac function significantly. Fig 6A and 6B demonstrated that the SM-HGF group had the highest values of LVSP and +dp/dt_max_ as compared to the SM-GFP and SM only groups. In addition, the SM-HGF group also exhibited the lowest values of LVEDP and–dp/dt_max_ (Fig 6C and 6D). These higher and lower values indicate a superior heart function in the SM-HGF group. Furthermore, the parameters LVSP and +dp/dt_max_ in the SM group were greater than the control group, indicating that the cell therapy exerts therapeutic benefits on MI.

The article "Transplantation of HGF gene-engineered skeletal myoblasts improve infarction recovery in a rat myocardial ischemia model" was retracted in 2023. Reasons: duplicated images; overlap with earlier publications; unreliable data; concerns about the images.

**Fig 6:** Implantation of HGF-modified skeletal myoblasts improves the heart function. The Ad-GFP or Ad-HGF transduced myoblasts were implanted into the myocardium in an MI model for 28 days. The cardiac functional parameters including LVSP (a) and +dp/dt_max_ (b), LVEDP (c), and dp/dt_min_ (d) were detected (n = 6, P<0.05, *P<0.05 *vs*. SM group; ^#^P<0.05 *vs*. SM-GFP group; ^†^P<0.05 *vs*. control group). (d) Western blot for Bcl-2 expression in SM transduced with Ad-HGF, vector control, and cell control group. (n = 6, P<0.05, *P<0.05 *vs*. SM group; ^#^P<0.05 *vs*. SM-GFP group; ^†^P<0.05 *vs*. control group).

### Implantation of HGF-transduced SM increases the vessel density and reduces fibrosis *in vivo*

Four weeks after cell transplantation, the size of the infarcted heart decreased and wall thickness increased in the SM-HGF group as compared to the SM,SM-GFP and control groups (sizes of the infarcted heart in SM-HGF *vs*. SM, SM-GFP, and control groups were 29.6 ± 3.2% *vs*. 37.8 ± 5.3%, 37.0 ± 4.9%, and 46.2 ± 3.6%, respectively; thicknesses of the cardiac wall were 2.12 ± 0.16 *vs*. 1.77 ± 0.32, 1.75 ± 0.21, and 1.22 ± 0.21, respetively; P<0.05, n = 6). The HGF group exhibited regional LV hypertrophy as measured by the LV border zone wall thickness, which was higher than SM, SM-GFP, and control groups (Fig 7A).

**Fig 7:** Implantation of HGF-modified skeletal myoblasts reduces infarct area and reduces collagen deposition. The Ad-GFP- or Ad-HGF-transduced myoblasts were implanted into the myocardium in an MI model for 28 days. (a) Representative images of histological sections in left ventricular stained with HE. Scale bars, 1 mm. (b) Images show that Sirius Red stained the cardiac sections from SM-GFP, SM only, SM-HGF group, and sham group, respectively. (c) The collagen volume fraction of SM-HGF group compared to the control group and SM group (n = 6, P<0.05, *P<0.05 vs. SM group; ^#^P<0.05 *vs*. SM-GFP group; ^†^P<0.05 *vs*. control group).

The collagen content in the non-infarcted area was stained by collagen-specific Sirius Red. The result showed that the collagen volume fraction significantly decreased in the SM-HGF group as compared to the SM-GFP and SM only groups. The combination of myocardial cell transplantation and HGF gene transfer markedly reduced the interstitial fibrosis in the non-infarcted myocardium (Fig 7B and 7C). The vascular density in the transplanted area was also evaluated and was found to increase significantly (P<0.05, n = 6/group) in the SM-HGF group as compared to the SM-GFP, SM only, and control groups (Fig 8A and 8B).

The article "Transplantation of HGF gene-engineered skeletal myoblasts improve infarction recovery in a rat myocardial ischemia model" was retracted in 2023. Reasons: duplicated images; overlap with earlier publications; unreliable data; concerns about the images.

**Fig 8:** Implantation of HGF-modified skeletal myoblasts increase the vessel density. The Ad-GFP- or Ad-HGF-transduced myoblasts were implanted into the myocardium in an MI model for 28 days. (a) Sections were stained with antibodies against Factor VIII to facilitate the counting of vessels. The representative images of the capillary density in transplanted area were shown. (b) The numbers of vascular densities of groups indicated (n = 6, P<0.05, *P<0.05 *vs*. SM group; ^#^P<0.05 *vs*. SM-GFP group; ^†^P<0.05 *vs*. control group).

## Discussion

In this study, we transduced the skeletal myoblasts with *HGF* gene using an adenovirus vector and evaluated the therapeutic effect of HGF-engineered cells in a rat MI model. The *HGF* gene transfer resulted in increased proliferation and survival of skeletal myoblasts *in vitro*. We confirmed that the implantation of HGF-modified skeletal myoblasts could improve the heart function by increasing the cell survival, inducing angiogenesis, and reducing fibrosis. Such combined therapeutics may overcome the current limitations of cell therapy and provide an alternative strategy for the treatment of patients with heart failure caused by MI.

The intramyocardial skeletal myoblast transplantation has been shown to improve the heart function after infarction in both experimental studies and clinical trials [29, 30]. Skeletal myoblasts are considered as the most promising cells for myocardial repair due to the high capacity of proliferation, secretion of angiogenic growth factors, and myogenic and contractile phenotypes. However, the engraftment efficiency of skeletal myoblasts is limited in the MI region owing to a high rate of mortality when implanted. The potential mechanisms underlying the limited engraftment efficiency of skeletal myoblasts in MI include the activation of pathways regulating apoptosis, inflammation, or immunological rejection. Several preconditioning methods including anti-apoptotic gene transfection and physiological pretreatment have been elucidated to enhance the survival of the grafted cells. The gene modification is speculated as the most efficient strategy for improving the engraftment of skeletal myoblasts in ischemic myocardium. Skeletal myoblasts were isolated and expanded from newborn SD rats and characterized for the expression of Desmin. The transfection efficiency of skeletal myoblasts using adenovirus vectors carrying the GFP gene was optimized. The Ad-HGF-transduced skeletal myoblasts secrete a high level of soluble HGF protein, which was maintained for a minimum of 2 weeks. These HGF gene-engineered skeletal myoblasts showed the enhanced capacity of proliferation and resistance to apoptosis *in vitro*. Furthermore, the transplantation of Ad-HGF-transduced skeletal myoblasts induces therapeutic angiogenesis, repopulates post-infarction scar, and improves the cardiac function in a rat MI model. We further confirmed that the engrafted cells or their progeny integrate with the host myocardium through the *Sry* gene that was used as a donor cell marker.

The article "Transplantation of HGF gene-engineered skeletal myoblasts improve infarction recovery in a rat myocardial ischemia model" was retracted in 2023. Reasons: duplicated images; overlap with earlier publications; unreliable data; concerns about the images.

Interestingly, the beneficial effects of skeletal myoblasts therapy may depend largely on their secretion of multiple growth factors. HGF is a multi-functional growth factor with anti-inflammatory and angiogenic activities [31]. Currently, clinical trials of the *HGF* gene therapy in the treatment of ischemic heart failure are ongoing [32]. Coupling the *HGF* gene therapy and cell therapy displayed a synergistic promoting effect on tissue regeneration and therapeutic angiogenesis. *HGF*-modified mesenchymal stem cells have been tested for the treatment of ischemic myocardium and radiation-induced lung and intestinal injury in animal models [14, 33, 34]. HGF modification also enhances the anti-arrhythmic properties of human bone marrow-derived mesenchymal stem cells [35]. Exogenous HGF stimulates the proliferation and inhibits the apoptosis of skeletal myoblasts via PI3K and p38 signals, downstream of the c-Met receptor [36]. These phenomena may be attributed to the overexpression of HGF in skeletal myoblasts that confers resistance to ischemia in MI. The results of our study also indicated that Ad-HGF-transfected myoblasts were capable of transient secretion of HGF both in culture and after cell transplantation into the myocardial scar tissue. Currently, both experimental and primary investigations confirm that *HGF* gene therapy and myoblasts therapy are effective in the treatment of ischemia-related diseases.

The transplantation of HGF-expressing skeletal myoblasts by adenovirus-mediated gene transfection results in high HGF expression within the rat myocardium suffering from acute infarction. This expression leads to a distinguished increase in LVSP and +dp/dt_max_, and a decrease in LVEDP and–dp/dt_max_, which is associated with improvement in ventricular remodeling and cardiac function, but without tumor formation. We further established that HGF-engineered skeletal myoblasts promote angiogenesis and enhance the survival of cardiomyocytes through the up-regulation of VEGF and Bcl-2 expression. HGF is known to induce VEGF-A expression in *in vitro* culture and promote angiogenesis through VEGF generation [28, 37]. Our data also confirmed that implantation of *HGF* gene-engineered skeletal myoblasts enhances the release of VEGF in the ischemic heart. The HGF-regulated VEGF expression was found to be involved in multiple pathways downstream of the c-Met receptor including PI3K/Akt, MAPK, and STAT3 [38]. Given the close relationship between vascular density and cell survival, the VEGF-mediated angiogenesis might contribute towards improved engraftment of HGF-transfected cells in failing heart, which could ameliorate the heart function post-MI. Moreover, HGF-induced cell survival was associated with the c-Met-Bcl-2-caspase-3 signaling pathways [39]. We found that the levels of Bcl-2 significantly increased in the myocardial tissue after cell transplantation. Bcl-2 plays crucial roles in the regulation of survival or death of myoblasts after cell transplantation. The overexpression of Bcl-2 enhanced the secretion of multiple angiogenic growth factors, such as VEGF, bFGF, and HGF [40]. The elevated level of Bcl-2 exerted a profound inhibitory effect on apoptosis and distinctly improved both cell survival and cardiac function. Thus, the anti-apoptotic effects of HGF might be mediated by Bcl-2 up-regulation.

The article "Transplantation of HGF gene-engineered skeletal myoblasts improve infarction recovery in a rat myocardial ischemia model" was retracted in 2023. Reasons: duplicated images; overlap with earlier publications; unreliable data; concerns about the images.

Nevertheless, the current study presents one limitation. Herein, the transplantation of *HGF*-engineered skeletal myoblasts improves the hemodynamic index. However, further studies using echocardiography are essential to determine the effect of engraftment of skeletal myoblasts on the changes in ejection fraction (EF) and cardiac output (CO).

In summary, we evaluated the therapeutic effect of *HGF* gene-engineered skeletal myoblasts on infarcted myocardium by enhancing angiogenesis, suppressing apoptosis, and reducing myocardial fibrosis. Thus, the transplantation of myoblasts combined with *HGF* gene therapy might be a promising strategy in the treatment of heart failure caused by MI.
